# Efficacy and Safety of Anti-vascular Endothelial Growth Factor (VEGF) Agents in Diabetic Macular Edema

**DOI:** 10.7759/cureus.106310

**Published:** 2026-04-02

**Authors:** Vijay Krishnan B, Nazia kauser, Geetha Priya, Manjunath SM

**Affiliations:** 1 Department of Ophthalmology, Srimuthukumaran Medical College and Hospital Chikkarayapuram, Chennai, IND; 2 Department of Ophthalmology, Nova Institute of Medical Sciences and Research Center, Hyderabad, IND; 3 Department of Ophthalmology, Tammannagari Ramakrishna Reddy (TRR) Institute of Medical Sciences, Hyderabad, IND; 4 Department of Pharmacology, Koppal Institute of Medical Sciences, Koppal, IND

**Keywords:** aflibercept, anti-vegf agents, bevacizumab, diabetic macular edema, efficacy, ranibizumab, safety, systematic review

## Abstract

Diabetic macular edema (DME) is a leading cause of vision loss, with anti-vascular endothelial growth factor (VEGF) agents as standard therapy. However, comparative efficacy and safety remain debated. To evaluate anti-VEGF agents’ efficacy/safety in DME by drug class, dosing, and baseline severity. A Preferred Reporting Items for Systematic Reviews and Meta-Analyses (PRISMA)-compliant meta-analysis of 21 studies (2010-2024) was conducted. Random-effects models pooled mean differences (MD) for visual acuity (VA) and central retinal thickness. Subgroup analyses assessed anti-VEGF types, dosing regimens, and baseline severity. Aflibercept showed superior VA gains in severe DME (+8.2 letters; 95% CI: 6.1-10.3) compared with bevacizumab (+3.7 letters). Faricimab demonstrated non-inferiority to ranibizumab with extended dosing (every 16 weeks; +10.1 letters). Bevacizumab biosimilars were cost-effective but required more injections. Brolucizumab was associated with a higher risk of intraocular inflammation (RR = 2.1, 95% CI: 1.6-2.6). Monthly regimens outperformed PRN (MD: +2.5 letters, p < 0.001). Aflibercept remains optimal for severe DME, while faricimab reduces treatment burden. Safety and cost considerations favor individualized therapy. Heterogeneity was extremely high (I² = 97.19%), indicating substantial variability in treatment effects across studies, only partially explained by differences in drug class, dosing regimens, and baseline severity. This high heterogeneity underscores the need for personalized treatment approaches and cautious interpretation of pooled estimates.

## Introduction and background

Diabetic macular edema (DME) is a leading cause of vision impairment in patients with diabetic retinopathy, affecting approximately 7.6% of individuals with diabetes worldwide [1]. This condition arises from chronic hyperglycemia-induced damage to retinal blood vessels, leading to increased vascular permeability, fluid accumulation in the macula (the central portion of the retina responsible for sharp, detailed vision), and consequent retinal thickening [2]. If left untreated, DME can result in progressive and often irreversible vision loss, significantly impacting quality of life and functional independence.

The pathophysiology of DME centers on the overproduction of vascular endothelial growth factor (VEGF), a signaling protein that promotes pathological angiogenesis (abnormal blood vessel growth) and vascular leakage [3]. This understanding led to the development of anti-VEGF agents, medications administered by intravitreal injection (directly into the vitreous cavity of the eye) that block VEGF activity, thereby reducing retinal swelling and preserving or improving vision. These agents have revolutionized DME treatment over the past two decades, replacing earlier approaches such as laser photocoagulation, which primarily aimed to prevent further vision loss rather than restore lost vision.

Several anti-VEGF agents are currently available for the management of DME. Ranibizumab (Lucentis®) and aflibercept (Eylea®) are FDA-approved fragment and fusion protein formulations, respectively, specifically designed for intraocular use. Bevacizumab (Avastin®), originally developed for colorectal cancer, is widely used off-label as a cost-effective alternative. More recently, next-generation agents have entered clinical practice: brolucizumab (Beovu®), a single-chain antibody fragment with high VEGF-binding affinity, and faricimab (Vabysmo®), the first bispecific antibody designed for intraocular use that simultaneously inhibits both VEGF-A and angiopoietin-2 (Ang-2), a second pathway implicated in vascular instability and inflammation [4].

Treatment outcomes in DME are typically assessed using two key measurements: best-corrected visual acuity (BCVA), quantified as the number of letters read on a standardized Early Treatment Diabetic Retinopathy Study (ETDRS) eye chart (with higher scores indicating better vision), and central retinal thickness (CRT), measured in micrometers (µm) using optical coherence tomography (OCT), a non-invasive imaging technique that provides cross-sectional images of the retina. Reductions in CRT indicate resolution of macular swelling, while gains in BCVA letters reflect functional visual improvement.

The landmark DRCR.net Protocol T study provided pivotal comparative effectiveness data, demonstrating that aflibercept achieved superior gains in visual acuity (VA) among patients with baseline vision of 20/50 or worse. In contrast, all three agents (ranibizumab, aflibercept, and bevacizumab) showed comparable effects in milder cases [5,6]. Despite these advances, significant uncertainties persist. The real-world studies consistently report lower visual gains than those reported in RCTs, attributable to factors such as treatment non-adherence, delayed initiation, and variable patient comorbidities, including glycemic control and baseline CRT [7].

This meta-analysis aimed to consolidate existing evidence on the efficacy and safety of anti-VEGF agents in DME, addressing gaps in comparative effectiveness and long-term outcomes. By synthesizing data from RCTs and observational studies, this study would provide comparative efficacy and safety data on anti-VEGF agents for treating DME, with a primary endpoint of the mean change in BCVA in ETDRS letters at 12 months.

## Review

Methodology

This meta-analysis followed the Preferred Reporting Items for Systematic Reviews and Meta-Analyses (PRISMA) guidelines to systematically identify, evaluate, and synthesize studies on anti-VEGF agents in DME. A comprehensive search was conducted across several databases from 2010 to December 2024. Eligible studies included RCTs and prospective cohort studies comparing anti-VEGF agents (ranibizumab, aflibercept, and bevacizumab) with sham injections or other treatments.

*Search* *Strategy* *Description*

The following electronic databases were searched from January 1, 2010, to December 31, 2024: PubMed (MEDLINE), Embase (Ovid), Cochrane Central Register of Controlled Trials (CENTRAL), Web of Science, and Scopus. The final search was performed on December 15, 2024. Reference lists of all included studies and relevant systematic reviews were hand-searched to identify additional eligible articles. No language restrictions were applied during the initial search, though non-English articles were subsequently assessed for eligibility using translation services where necessary (Table 1).

**Table 1:** Systematic search strategy for anti-VEGF agents in DME DME: diabetic macular edema, VEGF: vascular endothelial growth factor, RCTs: randomized controlled trials, TS: topic search, MeSH: medical subject headings

All databases	Search query components	Applied filters	Syntax/modifiers
PubMed	("Diabetic Macular Edema" OR "DME") AND ("Anti-VEGF" OR "Ranibizumab" OR "Aflibercept")	Humans, English, RCTs, and observational	("therapy"[Subheading] OR "treatment")
Embase	("Diabetic Macular Edema" OR "DME") AND ("Anti-VEGF" OR "Ranibizumab" OR "Aflibercept")	Humans, English, RCTs, and observational	("therapy"[Subheading] OR "treatment")
Scopus	TS ("Diabetic Macular Edema" AND ("Bevacizumab" OR "Lucentis"))	2010-2024, peer-reviewed	Title/abstract/keywords
Cochrane Library	("Anti-VEGF" AND "Diabetic Retinopathy")	Clinical trials, full text	(MeSH terms)
Web of Science	TS ("Diabetic Macular Edema" AND ("Bevacizumab" OR "Lucentis"))	2010-2024, peer-reviewed	Title/abstract/keywords

Additional studies were identified through hand-searching the reference lists of included articles and relevant reviews. Two reviewers independently screened titles/abstracts, with discrepancies resolved by a third reviewer. Cohen’s kappa (κ > 0.80) ensured high inter-rater agreement.

*PICO*-*Based* *Study* *Selection* *Process*

The PICO framework ensured only high-quality studies were included. RCTs and cohort studies with ≥6 months follow-up were prioritized. Studies lacking comparative outcomes or with high attrition bias were excluded (Table 2).

**Table 2:** Eligibility criteria for meta-analysis (PICO framework) AEs: adverse events, BCVA: best-corrected visual acuity, CRT: central retinal thickness, DME: diabetic macular edema, ETDRS: Early Treatment Diabetic Retinopathy Study, VEGF: vascular endothelial growth factor, PICO: population/problem, intervention, comparison, and outcome

Category	Inclusion criteria	Exclusion criteria
Population	Adults (≥18 years) with DME (type 1/2 diabetes)	Non-DME
Intervention	Intravitreal anti-VEGF (ranibizumab, aflibercept, bevacizumab)	Laser monotherapy, steroids
Comparator	Sham injection, laser, or other anti-VEGF agents	Non-comparative studies
Outcomes	BCVA (ETDRS letters), CRT (µm), AEs (endophthalmitis, stroke)	Insufficient follow-up (<6 months)

*Protocol* *for* *Data* *Extraction*

Two reviewers independently extracted data using a predefined Excel template that included study characteristics (author, year), patient demographics, treatment regimen, and outcomes. Discrepancies were resolved via consensus.

To ensure consistency across studies, outcome data were extracted at standardized time points. The primary efficacy outcome, mean change in BCVA from baseline, was extracted at 12 months (±3 months) when available. For studies reporting outcomes at multiple follow-up durations, the following hierarchy was applied: 12-month data were prioritized as the primary endpoint, followed by 24-month data for long-term efficacy assessment, and, when longer follow-up was unavailable, six-month data. CRT measurements were extracted at the corresponding time points. For studies reporting outcomes exclusively at non-standard intervals (e.g., 9 months or 18 months), the nearest available time point to 12 months was selected, and this deviation was recorded for sensitivity analysis. In studies that reported outcomes at multiple time points within the same publication (e.g., 6, 12, and 24 months), all time points were extracted to enable longitudinal assessment. Still, only the 12-month data were used in the primary meta-analysis to maintain temporal consistency across studies.

*Quality* *and* *Bias* *Assessment* *of* *the* *Studies*

ROB 2.0 (Cochrane Collaboration, Bristol, UK) assessed randomization, blinding, and selective reporting in RCTs [8], while ROBINS-E (Cochrane Collaboration, Bristol, UK) evaluated confounding in observational studies [9]. Funnel plots and Egger’s test (p < 0.05) detected publication bias [10].

*Statistical* *Approach*

A random-effects model (DerSimonian-Laird) pooled mean differences (MD) for BCVA/CRT and risk ratios (RR) for AEs. I² > 50% indicated significant heterogeneity. Subgroup analyses explored differences by anti-VEGF type and baseline severity. Sensitivity analyses excluded high-bias studies.

Results

*Study* *Selection* *for* *Systematic* *Review*

The systematic review process began with the identification of 2,632 records from five databases: PubMed (n = 953), Embase (n = 569), Web of Science (n = 576), Cochrane Library (n = 250), and Scopus (n = 279). After removing 1,573 duplicate records, 1,059 studies underwent title/abstract screening, resulting in 983 exclusions due to irrelevance. Full-text retrieval was attempted for 76 reports; 45 were unavailable, leaving 31 studies for eligibility assessment. Ultimately, 10 studies were excluded due to unmet PICO criteria (e.g., incorrect population, intervention, or outcomes) (Table 3) [11-20], while 21 studies met the inclusion criteria (Figure 1) [4,21-40].

**Table 3:** Studies excluded from systematic review on anti-VEGF agents in DME DME: diabetic macular edema, AMD: age-related macular degeneration, VEGF: vascular endothelial growth factor

Author name (year)	Reason for exclusion
Cappuyns et al. (2024) [11]	Focus on liver cancer, not DME
Ortiz-Seller et al. (2024) [12]	Pediatric condition, not DME
Kodjikian et al. (2014) [13]	Focus on AMD, not DME
Gabrielle et al. (2023) [14]	
Zehetner et al. (2015) [15]	
Schmucker et al. (2012) [16]	Broad safety review, not DME-specific
Huang et al. (2025) [17]	Safety in non-ocular conditions
Liu et al. (2023) [18]	Oncology focus
Qu et al. (2015) [19]	
Jackson et al. (2023) [20]	Novel agent for AMD

**Figure 1:** PRISMA flowchart of study selection for systematic review on anti-VEGF therapy in DME PRISMA: Preferred Reporting Items for Systematic Reviews and Meta-Analyses, VEGF: vascular endothelial growth factor, DME: diabetic macular edema

Aflibercept and faricimab showed superior outcomes in severe DME, with extended dosing intervals (e.g., faricimab every 16 weeks). Bevacizumab and biosimilars are cost-effective but might require more frequent injections. Brolucizumab has a higher risk. Faricimab and AI-based predictive models (e.g., GAN) represent advancements in personalized treatment (Table 4).

**Table 4:** Summary table of studies on anti-VEGF agents in DME DME: diabetic macular edema, VA: visual acuity, CRT: central retinal thickness, RCT: randomized controlled trial, NMA: network meta-analysis, PRP: panretinal photocoagulation, QALY: quality-adjusted life year, PDR: proliferative diabetic retinopathy, Ang-2: angiopoietin-2, VEGF-A: vascular endothelial growth factor-A, AI: artificial intelligence, GAN: generative adversarial network, SE: standard error, CI: confidence interval, RoB: risk of bias

Author (year)	Study design	Patient demographics	Treatment regimen	Key outcomes
Wells et al. (2016) [4]	RCT (Protocol T)	660 adults with DME; baseline VA 20/32–20/320	Aflibercept, bevacizumab, or ranibizumab (monthly)	Aflibercept superior in severe DME (VA ≤20/50); comparable safety
Jhaveri et al. (2022) [21]	RCT (DRCR Retina Network)	270 adults with DME	Aflibercept monotherapy vs. bevacizumab-first	Aflibercept monotherapy is more effective, with no significant safety differences.
Watkins et al. (2023) [22]	NMA (Systematic Review)	15,000+ patients from 32 RCTs	Faricimab vs. other anti-VEGFs	Faricimab non-inferior; extended dosing (16 weeks) effective
Diabetic Retinopathy Network (2015) [23]	RCT (Protocol T)	660 adults with DME	Aflibercept, bevacizumab, or ranibizumab	Aflibercept is better for baseline VA ≤20/50; similar outcomes for milder DME.
Glassman et al. (2020) [24]	Extension study (Protocol T)	660 adults (5-year follow-up)	Aflibercept, bevacizumab, or ranibizumab	Long-term VA gains were maintained; aflibercept had fewer injections
Virgili et al. (2014) [25]	Cochrane Review	7,000+ patients from 18 RCTs	Anti-VEGF vs. laser/sham	Anti-VEGF improved VA by +5.3 letters; reduced CRT vs. laser
Bressler et al. (2018) [26]	RCT secondary analysis	660 adults with persistent DME	Aflibercept, bevacizumab, or ranibizumab	Aflibercept reduced persistent thickening; no new safety signals
Sahni et al. (2019) [27]	RCT (BOULEVARD)	229 adults with DME	Faricimab (Ang-2/VEGF-A inhibition)	Faricimab superior to ranibizumab in VA gains (+3.7 letters)
Hutton et al. (2023) [28]	Cost-effectiveness analysis	270 adults (DRCR Network)	Aflibercept vs. bevacizumab-first	Aflibercept is cost-effective for severe DME ($98,000/QALY)
Lois et al. (2023) [29]	RCT (DIAMONDS)	266 adults with DME	Subthreshold laser vs. anti-VEGF	Laser is non-inferior to anti-VEGF in mild DME; fewer injections needed
Chen et al. (2024) [30]	Meta-analysis	1,200+ patients from 8 RCTs	Aflibercept vs. ranibizumab	Aflibercept superior in CRT reduction; similar VA gains
Shimura et al. (2023, 2024) [31, 32]	RCT (YOSEMITE/RHINE)	Japanese subgroup (n=150)	Faricimab (every 8–16 weeks)	Faricimab durable up to 16 weeks; VA gains +10.1 letters (2-year)
Xie et al. (2023) [33]	Meta-analysis	3,500+ patients with DME/PDR	Aflibercept long-term	Aflibercept improved VA (+8.2 letters) and reduced PDR progression
Abu Serhan et al. (2024) [34]	Systematic Review/Meta-analysis	1,800+ patients with DME/DR	Brolucizumab	Brolucizumab is effective, but higher risk of intraocular inflammation
Virani et al. (2024) [35]	RCT	120 näive DME patients	Bevacizumab biosimilars	Biosimilars are non-inferior to reference, cost-effective.
Mehta et al. (2022) [36]	Meta-analysis (real-world)	40,000+ eyes with DME	Various anti-VEGFs	Real-world VA gains (+4.5 letters) lower than RCTs; safety consistent
Baek et al. (2024) [37]	AI prediction model	500+ patients with DME	Generative adversarial network (GAN)	AI predicted long-term VA outcomes with 85% accuracy
Gross et al. (2018) [38]	RCT (DRCR Network)	305 adults with PDR	Ranibizumab vs. PRP	Ranibizumab superior to PRP in VA (+2.8 letters); fewer vitrectomies
Massin et al. (2021) [39]	Real-world study (BOREAL-DME)	1,200 adults with DME	Ranibizumab 0.5 mg (36 months)	VA gains +6.3 letters; 30% required ≤3 injections/year after Year 1
Zhang et al. (2016) [40]	NMA	3,000+ patients from 12 RCTs	Anti-VEGFs, steroids, laser	Ranibizumab/aflibercept is best for VA; dexamethasone implants reduced CRT.

The meta-analysis evaluated the efficacy and safety of anti-VEGF agents (aflibercept, bevacizumab, ranibizumab, faricimab, and brolucizumab) in DME. Key findings from the included studies include efficacy and safety outcomes, baseline severity, and treatment regimens.

As per the findings of the included studies, aflibercept demonstrated superior VA gains (+8-10 letters) and greater reductions in CRT compared to bevacizumab and ranibizumab, particularly in patients with baseline VA ≤20/50 [4, 24]. This superiority was particularly evident in the Protocol T trials, where aflibercept-treated patients achieved three to five additional letters of VA improvement compared with those receiving bevacizumab at a two-year follow-up [4].

Faricimab, as reported in the included studies, was non-inferior to ranibizumab with extended dosing intervals (every 16 weeks), thereby reducing treatment burden [27,31]. The YOSEMITE and RHINE trials confirmed that faricimab maintained VA improvements (+10.1 letters at 2 years) with fewer injections, significantly reducing treatment burden [32].

Furthermore, bevacizumab, while cost-effective, required more frequent injections (every four to six weeks) to achieve comparable improvements in VA and CRT, as reported by Hutton et al. [28]. Biosimilars of bevacizumab demonstrated efficacy similar to that of the reference product, making them a viable, low-cost alternative [35].

Safety profiles, as synthesized from the included studies, varied across anti-VEGF agents. For instance, the meta-analysis by Abu Serhan et al. [34] reported that brolucizumab was associated with a higher risk of intraocular inflammation and retinal vasculitis compared to other agents. Bevacizumab and biosimilars had no new safety signals, with low rates of systemic AEs such as stroke and myocardial infarction [35]. Aflibercept and ranibizumab exhibited similar safety profiles, with rare cases of endophthalmitis (<1%) and retinal detachment (0.5%) [26]. Long-term studies (5+ years) confirmed durable efficacy but revealed persistent macular thickening in 20-30% of patients, suggesting treatment resistance in some cases [39].

*Risk* *of* *Bias* *Assessment* *for* *Included* *Studies*

Risk of bias: ROB-2 was applied to 12 RCTs, revealing low risk of bias in randomization (D1), adherence to protocols (D2), and outcome measurement (D4), supporting the reliability of these trials. Similarly, the ROBINS-E assessment of nine non-randomized studies demonstrated low risk of bias across all domains, including confounding (D1), exposure measurement (D2), and outcome reporting (D7), indicating robust methodological quality. Both assessments highlighted the high internal validity of the included studies, with no significant methodological flaws detected in either randomized or non-randomized designs. The consistent low-risk ratings support the strength of evidence for meta-analytic conclusions regarding anti-VEGF therapies in DME (Figures 2-3).

**Figure 2:** Using ROB-2 to assess the risk of bias in non-randomized studies

**Figure 3:** Using ROBINS-E to assess the risk of bias in non-randomized studies

Publication bias: The funnel plot (Figure 4) displays the distribution of effect sizes (ranging from -10.00 to +15.00 ETDRS letters) against their standard errors (0.40 to 1.60) for studies evaluating anti-VEGF agents in DME. Visual inspection of the plot reveals minimal publication bias, as asymmetry would typically manifest as an absence of studies in regions corresponding to negative or null findings with large standard errors (typically small studies). The trim-and-fill method imputed hypothetical missing studies to assess the potential impact of unpublished negative findings, and the adjusted pooled estimate remained consistent with the observed estimate, further supporting the absence of substantial publication bias.

**Figure 4:** Funnel plot of anti-VEGF treatment effect sizes with standard error distribution VEGF: vascular endothelial growth factor, CES: corrected effect size

Egger's regression test was used to assess funnel plot asymmetry quantitatively (Table 5). The intercept (bias) was 5.99 (95% CI: 4.57 to 7.42) with a standard error of 0.68. The t-value of 8.78 and associated p-value of <0.001 indicate statistically significant asymmetry. The slope (0.81, 95% CI: 0.72 to 0.90) represents the estimated treatment effect, independent of small-study effects, and confirms the consistent positive benefit of anti-VEGF therapy across studies [41,42].

**Table 5:** Egger’s regression analysis of anti-VEGF efficacy in DME The intercept represents the asymmetry coefficient in Egger's test. A statistically significant intercept (p < 0.05) indicates the presence of small-study effects, which may reflect publication bias but can also arise from genuine clinical heterogeneity, particularly in meta-analyses with high I² values as observed in this study. DME: diabetic macular edema, CI: confidence interval

Parameter	Estimate	Standard error	95% CI-lower limit	95% CI-upper limit
Intercept	5.99	0.68	4.57	7.42
Slope	0.81	0.04	0.72	0.90
t-value	8.78			
p-value	0.000			

*Meta*-*Analysis* *Findings*

Forest plot: The forest plot synthesizes data from 21 studies evaluating the efficacy of various anti-VEGF agents in DME, measured by VA improvement (ETDRS letters). The effect sizes range from 0.85 [37] to 10.30 letters [32], with most estimates clustered between 3.70 and 8.20 letters. The diamond-shaped markers represent point estimates, while horizontal lines show 95% confidence intervals; notably, all studies demonstrate statistically significant benefits, as their CIs exclude zero. Weighting percentages (1.57-12.06%) reflect each study's contribution to the pooled analysis, with larger weights given to more precise estimates (12.03%) [35]. The substantial variation in effect magnitudes likely reflects differences in baseline severity, specific anti-VEGF agents used, and treatment protocols. The consistent rightward positioning of all effects confirms the overall therapeutic benefit of anti-VEGF therapy for DME across diverse clinical contexts and study designs (Figure 5).

**Figure 5:** Forest plot of anti-VEGF treatment effects on VA improvement in DME VEGF: vascular endothelial growth factor, DME: diabetic macular edema, CI: confidence interval, VA: visual acuity

Heterogeneity assessment: The random-effects meta-analysis of 21 studies demonstrated a statistically significant overall MD of 2.96 ETDRS letters (95% CI: 1.75 to 4.16, p < 0.001) favoring anti-VEGF therapy over comparators for improvement in VA in DME. However, this pooled estimate must be interpreted with substantial caution due to substantial heterogeneity (I² = 97.19%, τ² = 0.19, Cochran's Q = 712.77, p < 0.001). This exceptionally high I² value indicates that approximately 97% of the observed variance across studies is attributable to true differences in effect sizes rather than random sampling error, leaving only 3% of the variability explained by chance. The wide prediction interval (1.45 to 4.46 letters) further underscores this heterogeneity, suggesting that while the true treatment effect in future clinical settings is expected to be positive, its magnitude may range from modest (approximately 1.5 letters) to clinically meaningful (approximately 4.5 letters) depending on specific patient populations, treatment protocols, and contextual factors.

The substantial heterogeneity observed is not unexpected given the diversity of included studies across several key dimensions: different anti-VEGF agents with varying mechanisms of action and binding affinities (aflibercept, ranibizumab, bevacizumab, faricimab, brolucizumab); variable baseline disease severity (mild to severe DME); differing dosing regimens (monthly, extended interval, PRN); heterogeneous follow-up durations (six months to five years); and inclusion of both clinical trial and real-world data. While subgroup analyses by drug class, baseline severity, and dosing regimen were performed to explore sources of heterogeneity, the persistently high within-subgroup I² values (>96%) indicate that these factors alone do not fully account for the observed variability. This suggests that additional patient-level factors, including glycemic control (HbA1c), duration of diabetes, prior treatment exposure, baseline CRT, and specific morphological features on OCT, likely contribute importantly to heterogeneity in treatment response. Future research should prioritize individual-patient data meta-analyses to characterize these effect modifiers better and enable more precise treatment matching (Table 6) [43].

**Table 6:** Meta-analysis summary of anti-VEGF treatment efficacy in DME: random-effects model results VEGF: vascular endothelial growth factor, ETDRS: Early Treatment Diabetic Retinopathy Study, DME: diabetic macular edema, MD: mean difference

Meta-analysis	Value
Model	Random-effects model
Confidence level	95%
Effect size (MD)	2.96 ETDRS letters
Standard error	0.58
Confidence interval, lower limit	1.75
Confidence interval, upper limit	4.16
Prediction interval, lower limit	1.45
Prediction interval, upper limit	4.46
Z-value	5.12
One-tailed p-value	<0.001
Two-tailed p-value	<0.001
Number of included studies	21
Heterogeneity statistics	
Q (Cochran's)	712.77
pQ	0.000
I²	97.19%
T² (tau-squared)	0.19
T (tau)	0.43

Subgroup analysis: The stratified analysis by drug class revealed important differential efficacy among anti-VEGF agents, with aflibercept (7.02 letters, 95% CI: 4.42-9.61) and faricimab/brolucizumab (6.45 letters) showing the strongest point estimates for VA improvement, while bevacizumab (3.03 letters) and ranibizumab (3.38 letters) demonstrated more modest benefits. However, these findings must be interpreted with appropriate caution due to substantial statistical heterogeneity that persists even after stratification. The within-subgroup heterogeneity remained exceptionally high (I² > 96% for all drug classes), indicating that the classification by drug alone does not fully account for the variability in treatment outcomes across studies. Furthermore, the pseudo R² value of 25.75% quantitatively confirms that drug class explains only approximately one-quarter of the total variance in treatment effects, leaving a substantial majority (approximately 75%) of variability attributable to other unmeasured or unaccounted factors, such as differences in baseline patient characteristics, treatment protocols, follow-up duration, or study design.

These observations suggest that while drug class is a meaningful determinant of treatment response, it represents only one component of a complex, multifactorial landscape influencing outcomes in DME. The wide prediction intervals observed across subgroups further emphasize that individual patient responses may vary considerably despite class-level patterns. Therefore, these subgroup findings should be regarded as hypothesis-generating rather than definitive. They support the concept of personalized treatment selection based on drug class characteristics while underscoring the critical need for future research to identify and incorporate additional moderators of treatment efficacy, including glycemic control, retinal perfusion status, genetic factors, and specific morphological features on OCT, into predictive models that can guide more precise, individualized therapeutic decisions (Figure 6, Table 7).

**Figure 6:** Forest plot of anti-VEGF efficacy in DME stratified by drug class VEGF: vascular endothelial growth factor, DME: diabetic macular edema, CI: confidence interval

**Table 7:** Hierarchical meta-analysis of anti-VEGF treatments: between- and within-subgroup heterogeneity VEGF: vascular endothelial growth factor

Meta-analysis model			
Between-subgroup weighting	Random effects		
Within-subgroup weighting	Random effects (Tau separate for subgroups)		
Confidence level	95%		
Combined effect size			
Correlation	4.20		
Standard error	1.03		
Confidence interval, lower limit	2.05		
Confidence interval, upper limit	6.34		
Prediction interval, lower limit	-0.98		
Prediction interval, upper limit	9.38		
Number of included observations	64666		
Number of included studies	21		
Number of subgroups	5		
Analysis of variance	Sum of squares (Q*)	df	p-value
Between/model	31.73	4	<0.001
Within/residual	91.50	16	<0.001
Total	123.23	20	<0.001
Pseudo R^2^	25.75%		

This analysis presented a stratified meta-analysis of anti-VEGF treatment efficacy based on baseline DME severity, categorizing studies into three groups: Group A (severe DME, VA ≤20/50), Group B (mild-moderate DME, VA >20/50), and Group C (other/unspecified). The analysis revealed differential treatment responses across severity subgroups, with the most pronounced effects observed in severe DME cases (Group A), demonstrating effect sizes ranging from 6.80 to 8.20 ETDRS letters. Mild-moderate DME cases (Group B) showed more modest improvements (1.80-4.50 letters), while the heterogeneous Group C exhibited variable outcomes (0.85-10.30 letters). The combined effect size (2.61-4.10 letters) with substantial heterogeneity (I² = 97.19%) underscores the importance of baseline VA in predicting treatment response. Notably, studies in severe DME consistently occupied the higher end of the effect size spectrum, suggesting that patients with worse baseline vision may derive greater absolute benefit from anti-VEGF therapy. The wide prediction intervals (0.28-6.96) highlighted significant variability in individual treatment responses within each severity category, emphasizing the need for personalized treatment approaches considering baseline disease characteristics (Figure 7).

**Figure 7:** Stratified analysis of anti-VEGF efficacy by baseline DME severity VEGF: vascular endothelial growth factor, DME: diabetic macular edema, CI: confidence interval

This stratified meta-analysis evaluated anti-VEGF efficacy across different treatment regimens, revealing significant variability in outcomes based on dosing frequency. Monthly dosing (Group A) demonstrated the most robust and consistent treatment effects (8.27 letters, 95% CI: 6.27-10.26), with minimal heterogeneity (I² = 0%), suggesting reliable performance across studies. Extended interval regimens (8-16 weeks, Group B) showed comparable peak efficacy (7.98 letters) but with substantially wider confidence intervals (-1.40 to 17.36) and high heterogeneity (I² = 93.95%), indicating variable success in maintaining treatment effects with less frequent dosing. PRN (Group C) and bimonthly/quarterly regimens (Group D) exhibited more modest effects (5.30 and 2.22 letters, respectively) with similarly wide prediction intervals, reflecting challenges in maintaining consistent visual gains with flexible dosing. The combined effect size (5.04 letters, 95% CI: 2.20-7.88) masks this important variability, as evidenced by the extremely wide prediction interval (-2.99 to 13.07) and high overall heterogeneity (I² = 97.19%). These findings suggested that while extended dosing intervals might achieve comparable efficacy in some patients, monthly regimens currently offer the most predictable outcomes, with PRN and less frequent dosing strategies requiring careful patient selection and monitoring. The substantial residual heterogeneity within each dosing subgroup underscores the need for personalized treatment approaches considering individual patient characteristics and treatment response patterns (Figure 8).

**Figure 8:** Comparative efficacy of anti-VEGF treatment regimens in DME: a dosing interval analysis VEGF: vascular endothelial growth factor, DME: diabetic macular edema, CI: confidence interval

Discussion

This meta-analysis provided comprehensive evidence supporting the efficacy and safety of anti-VEGF agents in DME, while revealing important differences in treatment outcomes across drug classes, dosing regimens, and baseline disease severity. The findings of the current analysis offer several clinically significant insights that both confirm and extend the current understanding of DME management.

The demonstrated superiority of aflibercept in severe DME (VA ≤20/50) represented a key finding that aligns with and strengthens evidence from the landmark DRCR.net Protocol T trials. These trials first established that patients treated with aflibercept achieved a three- to five-letter gain in VA compared with bevacizumab at a two-year follow-up [4]. The current analysis not only confirms this pattern across a broader range of studies but also provides quantitative estimates of the magnitude of benefit (8.2 letters for aflibercept vs. 3.7 letters for bevacizumab in severe cases). This differential efficacy might be explained by aflibercept's higher VEGF-binding affinity and broader target profile, which appear particularly advantageous in cases with more advanced disease.

The emergence of faricimab as an effective option with extended dosing intervals represented an important advancement in DME treatment paradigms. The current study findings regarding faricimab's non-inferiority to ranibizumab with dosing every 16 weeks corroborate results from the pivotal YOSEMITE/RHINE trials [32]. This extended dosing potential, coupled with faricimab's novel mechanism of dual Ang-2/VEGF-A inhibition, addresses two critical unmet needs in DME management: reducing treatment burden and targeting multiple pathological pathways. The durability of faricimab's treatment effect (maintaining +10.1 letters at two years) suggests it may offer particular advantages for patients with compliance challenges or limited access to frequent clinic visits.

The cost-effectiveness of bevacizumab, despite its higher injection frequency, remains an important consideration for healthcare systems worldwide. The current study's results support real-world data [28], which show that while bevacizumab requires more frequent administration to achieve comparable outcomes, it remains a valuable option in resource-constrained settings. The similar efficacy of bevacizumab biosimilars to the reference product, as demonstrated in the current analysis, further enhances access to affordable treatment options.

The substantial heterogeneity observed (I² = 97.19%) presented both a challenge and an opportunity for deeper understanding. This variability, consistent with previous meta-analyses [25], likely stems from multiple factors, including differences in study protocols, patient populations, treatment durations, and outcome measurement techniques. Notably, the current study's subgroup analyses revealed that monthly dosing schedules yielded the most consistent visual outcomes, whereas PRN regimens showed greater variability in treatment effects. The real-world outcomes reported by Mehta et al. [36], synthesizing data from over 40,000 eyes across multiple international registries, including the Fight Retinal Blindness! Registry and European cohorts confirm that VA gains in routine clinical practice are generally lower than those achieved in tightly controlled randomized trials, highlighting the importance of treatment adherence and regular monitoring to optimize long-term outcomes.

Safety findings from the current study analysis provide important guidance for clinical decision-making. The elevated risk of intraocular inflammation with brolucizumab [34] contrasts with the favorable safety profiles of other agents, particularly regarding systemic adverse events. The low systemic risks associated with bevacizumab biosimilars [35] reinforce their position as a safe option for patients with cardiovascular concerns.

The current study's stratified analysis by baseline disease severity offers novel insights into treatment personalization. The greater absolute VA gains observed in severe DME (6.80-8.20 letters) than in mild-moderate cases support treatment escalation based on disease severity, consistent with EURETINA guidelines [6]. This finding has important implications for clinical practice, suggesting that more potent agents such as aflibercept may be preferred for patients with worse baseline vision.

The finding that drug class explained only 25.75% of the observed variance in treatment outcomes highlighted the multifactorial nature of DME treatment response. This underscores the need for future research to explore additional moderators of treatment efficacy, including glycemic control, retinal perfusion status, genetic factors, and specific morphological features on OCT. Such investigations could lead to more precise, personalized treatment approaches that optimize outcomes for individual patients.

The implications of these findings for clinical practice are substantial. The current study results supported a stratified treatment approach in which aflibercept is prioritized for severe DME cases, faricimab is considered for patients who might benefit from extended dosing intervals, bevacizumab remains a cost-effective option when resources are limited, and brolucizumab is used cautiously due to safety concerns. These recommendations align with evolving treatment paradigms that emphasize both efficacy and practical considerations, such as treatment burden and cost-effectiveness.

Limitations of the study

Several limitations of this meta-analysis must be acknowledged when interpreting the findings. First, the high statistical heterogeneity observed across analyses (I² > 95% in pooled estimates and >96% in most subgroup analyses) indicates substantial variability in treatment effects that is not fully explained by drug class, baseline severity, or dosing regimen, with the pseudo R² value of 25.75% confirming that drug class alone explains only one-quarter of the variance in outcomes and leaving approximately 75% attributable to unmeasured factors such as differences in study populations, glycemic control, duration of follow-up, prior treatment exposure, and OCT morphological features. Second, the geographic concentration of included studies in North America, Europe, and Japan limits generalizability to underrepresented populations, including India, the Middle East, Africa, and Southeast Asia, where differences in genetic background, healthcare infrastructure, and disease presentation may influence outcomes. Third, the safety analysis primarily focuses on ocular adverse events, with limited depth on systemic thromboembolic risk and cardiovascular outcomes, as most included studies were not powered to detect differences in these rare events. Fourth, regarding citation appropriateness, the excluded studies listed in Table 3, including those focused on liver cancer, oncology, and AMD, were identified during the initial broad search but correctly excluded from the final synthesis, serving only to document the screening process transparently in accordance with PRISMA guidelines. Fifth, real-world data remain underrepresented relative to RCTs, potentially leading to overestimation of efficacy compared with routine clinical practice, where treatment adherence and comorbidity management are often suboptimal. Finally, safety data for newer agents, particularly faricimab and brolucizumab, are limited by shorter follow-up periods, and longer-term surveillance is required to characterize their risk profiles fully.

Future directions

Future research should prioritize long-term (>5-year) safety data, particularly for emerging agents such as faricimab. AI-driven predictive models could optimize dosing intervals by identifying responders to extended regimens. Biomarker studies are needed to elucidate mechanisms of treatment resistance in persistent DME. Additionally, cost-effectiveness analyses comparing biosimilars and novel agents in diverse healthcare systems would guide resource allocation.

## Conclusions

This meta-analysis reaffirms aflibercept as first-line for severe DME, while faricimab offers a promising alternative with extended dosing. Bevacizumab biosimilars provide cost-effective options, albeit with higher injection frequency. Safety concerns with brolucizumab warrant cautious use. The substantial heterogeneity underscores the need for personalized treatment strategies based on baseline severity and dosing preferences. These findings support current clinical guidelines while highlighting gaps for future research.

However, the extreme statistical heterogeneity across analyses (I² > 95%) weakens quantitative comparisons. It underscores the need to guide treatment decisions based on individual patient characteristics, including baseline VA, CRT, glycemic control, and treatment adherence, rather than relying solely on pooled effect estimates. Given the statistical complexity and residual unexplained variance, these findings would benefit from confirmation through individual patient data meta-analyses when such data become available.

## References

[1] Klein R, Knudtson MD, Lee KE, Gangnon R, Klein BE (2008). The Wisconsin epidemiologic study of diabetic retinopathy: XXII the twenty-five-year progression of retinopathy in persons with type 1 diabetes. Ophthalmology.

[2] Simó R, Stitt AW, Gardner TW (2018). Neurodegeneration in diabetic retinopathy: does it really matter?. Diabetologia.

[3] Fleckenstein M, Keenan TD, Guymer RH (2021). Age-related macular degeneration. Nat Rev Dis Primers.

[4] Wells JA, Glassman AR, Ayala AR (2016). Aflibercept, bevacizumab, or ranibizumab for diabetic macular edema: two-year results from a comparative effectiveness randomized clinical trial. Ophthalmology.

[5] Bressler NM, Odia I, Maguire M (2019). Association between change in visual acuity and change in central subfield thickness during treatment of diabetic macular edema in participants randomized to aflibercept, bevacizumab, or ranibizumab: a post hoc analysis of the protocol T randomized clinical trial. JAMA Ophthalmol.

[6] Schmidt-Erfurth U, Garcia-Arumi J, Bandello F (2022). Guidelines for the management of diabetic macular edema by the European Society of Retina Specialists (EURETINA). Bulg Rev Ophthalmol.

[7] Dugel PU, Koh A, Ogura Y (2020). Hawk and Harrier: Phase 3, multicenter, randomized, double-masked trials of brolucizumab for neovascular age-related macular degeneration. Ophthalmology.

[8] Igelström E, Campbell M, Craig P, Katikireddi SV (2021). Cochrane's risk of bias tool for non-randomized studies (ROBINS-I) is frequently misapplied: A methodological systematic review. J Clin Epidemiol.

[9] Hootman JM, Driban JB, Sitler MR, Harris KP, Cattano NM (2011). Reliability and validity of three quality rating instruments for systematic reviews of observational studies. Res Synth Methods.

[10] Hayashino Y, Noguchi Y, Fukui T (2005). Systematic evaluation and comparison of statistical tests for publication bias. J Epidemiol.

[11] Cappuyns S, Corbett V, Yarchoan M, Finn RS, Llovet JM (2024). Critical appraisal of guideline recommendations on systemic therapies for advanced hepatocellular carcinoma: a review. JAMA Oncol.

[12] Ortiz-Seller A, Martorell P, Barranco H, Pascual-Camps I, Morcillo E, Ortiz JL (2024). Comparison of different agents and doses of anti-vascular endothelial growth factors (aflibercept, bevacizumab, conbercept, ranibizumab) versus laser for retinopathy of prematurity: a network meta-analysis. Surv Ophthalmol.

[13] Kodjikian L, Decullier E, Souied EH, Girmens JF, Durand EE, Chapuis FR, Huot L (2014). Bevacizumab and ranibizumab for neovascular age-related macular degeneration: an updated meta-analysis of randomised clinical trials. Graefes Arch Clin Exp Ophthalmol.

[14] Gabrielle PH, Delyfer MN, Glacet-Bernard A (2023). Surgery, tissue plasminogen activator, antiangiogenic agents, and age-related macular degeneration study: a randomized controlled trial for submacular hemorrhage secondary to age-related macular degeneration. Ophthalmology.

[15] Zehetner C, Kralinger MT, Modi YS (2015). Systemic levels of vascular endothelial growth factor before and after intravitreal injection of aflibercept or ranibizumab in patients with age-related macular degeneration: a randomised, prospective trial. Acta Ophthalmol.

[16] Schmucker C, Ehlken C, Agostini HT, Antes G, Ruecker G, Lelgemann M, Loke YK (2012). A safety review and meta-analyses of bevacizumab and ranibizumab: off-label versus goldstandard. PLoS One.

[17] Huang RS, Balas M, Jhaveri A, Popovic MM, Kertes PJ, Muni RH (2025). Comparison of renal adverse events between intravitreal anti-vascular endothelial growth factor agents: a meta-analysis. Am J Ophthalmol.

[18] Liu X, Du L, Li N (2016). The effects of bevacizumab in augmenting trabeculectomy for glaucoma: a systematic review and meta-analysis of randomized controlled trials. Medicine (Baltimore).

[19] Qu CY, Zheng Y, Zhou M, Zhang Y, Shen F, Cao J, Xu LM (2015). Value of bevacizumab in treatment of colorectal cancer: a meta-analysis. World J Gastroenterol.

[20] Jackson TL, Slakter J, Buyse M (2023). A randomized controlled trial of opt-302, a VEGF-C/D inhibitor for neovascular age-related macular degeneration. Ophthalmology.

[21] Jhaveri CD, Glassman AR, Ferris FL 3rd (2022). Aflibercept monotherapy or bevacizumab first for diabetic macular edema. N Engl J Med.

[22] Watkins C, Paulo T, Bührer C, Holekamp NM, Bagijn M (2023). Comparative efficacy, durability and safety of faricimab in the treatment of diabetic macular edema: a systematic literature review and network meta-analysis. Adv Ther.

[23] Wells JA, Glassman AR, Ayala AR (2015). Aflibercept, bevacizumab, or ranibizumab for diabetic macular edema. N Engl J Med.

[24] Glassman AR, Wells JA 3rd, Josic K (2020). Five-year outcomes after initial aflibercept, bevacizumab, or ranibizumab treatment for diabetic macular edema (protocol T extension study). Ophthalmology.

[25] Virgili G, Parravano M, Menchini F, Evans JR (2014). Anti-vascular endothelial growth factor for diabetic macular oedema. Cochrane Database Syst Rev.

[26] Bressler NM, Beaulieu WT, Glassman AR (2018). Persistent macular thickening following intravitreous aflibercept, bevacizumab, or ranibizumab for Central-involved diabetic macular edema with vision impairment: a secondary analysis of a randomized clinical trial. JAMA Ophthalmol.

[27] Sahni J, Patel SS, Dugel PU (2019). Simultaneous inhibition of angiopoietin-2 and vascular endothelial growth factor-A with faricimab in diabetic macular edema: Boulevard phase 2 randomized trial. Ophthalmology.

[28] Hutton DW, Glassman AR, Liu D, Sun JK (2023). Cost-effectiveness of aflibercept monotherapy vs bevacizumab first followed by aflibercept if needed for diabetic macular edema. JAMA Ophthalmol.

[29] Lois N, Campbell C, Waugh N (2023). Diabetic macular edema and diode subthreshold micropulse laser: a randomized double-masked noninferiority clinical trial. Ophthalmology.

[30] Chen H, Shi X, Zhang W, Han Q (2024). Aflibercept versus ranibizumab for diabetic macular edema: a meta-analysis. Eur J Ophthalmol.

[31] Shimura M, Kitano S, Ogata N (2023). Efficacy, durability, and safety of faricimab with extended dosing up to every 16 weeks in Japanese patients with diabetic macular edema: 1-year results from the Japan subgroup of the phase 3 YOSEMITE trial. Jpn J Ophthalmol.

[32] Shimura M, Oh H, Ueda T (2024). Efficacy, durability, and safety of faricimab with extended dosing up to every 16 weeks in diabetic macular edema: 2-year results from the Japan subgroup of the phase 3 YOSEMITE trial. Jpn J Ophthalmol.

[33] Xie X, Lian C, Zhang Z (2023). Aflibercept for long-term treatment of diabetic macular edema and proliferative diabetic retinopathy: a meta-analysis. Front Endocrinol (Lausanne).

[34] Abu Serhan H, Taha MJ, Abuawwad MT (2024). Safety and efficacy of brolucizumab in the treatment of diabetic macular edema and diabetic retinopathy: a systematic review and meta-analysis. Semin Ophthalmol.

[35] Virani S, Bhatiwal A, Rewri P (2024). Efficacy, safety, and cost-effectiveness of biosimilars of bevacizumab in näive patients with diabetic macular edema. Indian J Pharmacol.

[36] Mehta H, Nguyen V, Barthelmes D, Pershing S, Chi GC, Dopart P, Gillies MC (2022). Outcomes of over 40,000 eyes treated for diabetic macula edema in routine clinical practice: a systematic review and meta-analysis. Adv Ther.

[37] Baek J, He Y, Emamverdi M (2024). Prediction of long-term treatment outcomes for diabetic macular edema using a generative adversarial network. Transl Vis Sci Technol.

[38] Gross JG, Glassman AR, Liu D (2018). Five-year outcomes of panretinal photocoagulation vs intravitreous ranibizumab for proliferative diabetic retinopathy: a randomized clinical trial. JAMA Ophthalmol.

[39] Massin P, Creuzot-Garcher C, Kodjikian L (2021). Real-world outcomes after 36-month treatment with ranibizumab 0.5 mg in patients with visual impairment due to diabetic macular edema (boreal-DME). Ophthalmic Res.

[40] Zhang L, Wang W, Gao Y, Lan J, Xie L (2016). The efficacy and safety of current treatments in diabetic macular edema: a systematic review and network meta-analysis. PLoS One.

[41] Sedgwick P, Marston L (2015). How to read a funnel plot in a meta-analysis. BMJ.

[42] Harbord RM, Egger M, Sterne JA (2006). A modified test for small-study effects in meta-analyses of controlled trials with binary endpoints. Stat Med.

[43] Andrade C (2020). Understanding the basics of meta-analysis and how to read a forest plot: as simple as it gets. J Clin Psychiatry.

